The article "A Rare Case of Chronic Appendicitis Superimposed on an Incarcerated de Garengeot Hernia Prospectively Identified on Computed Tomography" was retracted in 2018. Reasons: no approval from an author; concerns about the data; concerns about the results or conclusions.

# A Rare Case of Chronic Appendicitis Superimposed on an Incarcerated de Garengeot Hernia Prospectively Identified on Computed Tomography

**DOI:** 10.1155/2018/5324320

**Published:** 2018-06-20

**Authors:** Alyssa Goldbach, Partha Hota, Andrew Czulewicz, Christine Burgert-Lon, Omar Agosto

**Affiliations:** ^1^Division of Abdominal Imaging, Department of Radiology, Temple University Hospital, Philadelphia, PA, USA; ^2^Department of Pathology, Jeanes Hospital, Temple University Health System, Philadelphia, PA, USA

## Abstract

The de Garengeot hernia is an uncommon and potentially confounding pathologic process in which the appendix is contained within a femoral hernia. While typically a benign incidental finding, superimposed acute appendicitis is a rare but serious complication. Identification of this entity is crucial to patient management and ultimately outcome with imaging playing a critical role. Cross-sectional imaging, with either CT or MRI, should be performed in all cases of suspected incarcerated de Garengeot hernia to facilitate the appropriate diagnosis and surgical intervention. Herein, we present the fifth case of a prospective CT diagnosis of the de Garengeot hernia in a 61-year-old female who presented with an irreducible right femoral hernia. The patient underwent CT examination which demonstrated the appendix within the femoral hernia sac with an associated periappendiceal fluid collection. The patient was taken for emergent surgical intervention at which time the appendix was found within the hernia sac. The appendix was removed, the defect repaired, and ultimately the patient recovered well.

## 1. Introduction

In 2005, Akopian and Alexander first termed a femoral hernia containing the appendix the de Garengeot hernia (DGH) after French surgeon Rene de Garengeot, who is credited as the first to describe this entity in 1731 [1, 2]. To date, there are a total of fewer than 100 cases of DGH reported in literature with only 4 cases prospectively identifying the DGH prior to surgical intervention [1, 3–8]. DGHs are typically an incidental and unexpected finding discovered during femoral hernia repairs with an incidence in less than 1% of surgically treated hernias [4, 7]. The discovery of an acute inflamed appendix within the hernia sac, is even less likely, occurring in roughly 0.08–0.13% of symptomatic patients with this discrepancy likely secondary to the lack of preoperative imaging or misdiagnosis of an incarcerated femoral hernia [4, 7, 9, 10]. Given the increased risk of complications such as bowel ischemia, necrosis, perforation, abscess, and peritonitis in DGHs, early recognition is crucial to patient care [7]. We herein report a rare case of an incarcerated DGH with superimposed chronic appendicitis prospectively characterized by computed tomography (CT).

## 2. Case Report

A 61-year-old female with a past medical history of hypertension, HIV, and hepatitis C presented to our hospital with a 1-week history of right groin tenderness and a palpable lump in her right groin. The patient stated that the lump had been growing in size since its sudden appearance approximately 1 week prior. The patient denied fever, nausea, vomiting, or changes in her bowel habits. Physical examination of the right groin, demonstrated a minimally tender irreducible hernia without overlying skin changes. Laboratory values were within normal limits aside from a mildly elevated white blood cell count of 7700/*μ*L. A contrast-enhanced CT of the abdomen and pelvis was obtained for further evaluation which demonstrated a fat- and fluid-containing right femoral hernia (Figures 1 and 2). The appendix was located within the hernia sac with an associated fluid periappendiceal collection measuring 3.9 × 5.3 × 4.7 cm (AP × TV × CC). The margins of the appendix were thickened concerning for a possible acute on chronic appendicitis with periappendiceal abscess or mucocele. Subsequent surgical dissection of the hernia sac revealed a gelatinous coagulated fluid and an inflamed appendix with a mucocele at the tip. The appendix was resected and the femoral hernia was repaired. Given the large size of the defect, a large Proloop plug® was placed with an antibiotic vancomycin soak and stitched to the pubic tubercle. A histopathological examination of the appendix showed inflammatory changes including serosal congestion, edema, and fibrosis, consistent with chronic appendicitis with superimposed reactive features of hernia sac adipose tissue due to hernia incarceration (Figure 3).

The patient recovered well, without complications, and was discharged home one day postoperatively.

## 3. Discussion

Abdominal wall hernias occur secondary to a weakness in either the abdominal wall musculature or peritoneal fascia which allows for the projection of intraperitoneal contents through the defect. The inguinal region is predisposed to two types of hernias: inguinal and femoral. Femoral hernias account for 3% of all external hernias and occur within the femoral sheath, below the inguinal ligament [9]. Defined as the most medial compartment of the femoral sheath, the femoral canal is bordered anterosuperiorly by the inguinal ligament, medially by the lacunar ligament, laterally by the femoral vein, and posteriorly by the pectineal ligament [11]. Femoral hernias present with incarceration in about 50% of the cases and are at an increased risk of strangulation (5–20%) compared to other hernia types because of the narrow and rigid neck of the hernia sac [2, 4, 12]. Femoral hernias may contain a variety of tissues with hernias containing the omentum, bowel, and ovaries having been described in the literature [2]. An appendix located within the hernia sac, the DGH, is a much rarer and less well-understood entity.

The etiology of DGHs remains disputed. Hussein et al. and Sharma et al. suggested that during embryological development abnormal bowel rotation results in an atypical appendiceal attachment, thus the cecal appendix is able to migrate into a femoral hernia [13, 14]. Zissin and colleagues alternatively suggested that an anatomically large cecum could push the appendix in the femoral hernia [5, 13]. DGHs are more common in women (13 : 1 female predominance), in keeping with the overall female predominance of femoral hernias, due to the combination of lifestyle, mechanical stress, and pregnancy [11, 12]. Risk factors for DGH include a long pelvic appendix, abnormal embryological bowel rotation, and a large mobile cecum [12].

Typically, the DGH presents with symptoms of incarcerated or strangulated groin hernia. Patients often have a nonreducible groin lump that is usually painful and/or tender to palpation, with erythematous and sometimes edematous overlying skin. Signs of a systemic inflammatory response including fever and elevated white blood cell count are also common. While more unusual signs and symptoms of bowel obstruction or bowel ischemia have been reported, they are rare occurring in only 14% of patients [11, 13].

The herniated appendix can result in appendicitis and eventually perforation and abscess formation. In a retrospective review of NCBI PubMed literature utilizing the keywords “de Garengeot hernia,” “appendix in femoral hernia,” and “perforation” yielded 15 cases reported to date of a perforated appendix within a femoral hernia sac (Table 1). Theories for the development of superimposed appendicitis within a DGH include initial inflammation of the appendix in the peritoneum with resultant gradual migration into the hernia or migration into the hernia sac as the initial event and followed by inflammation secondary to incarceration or external compression [4, 13]. Given the high incidence of femoral hernia strangulation, clinical symptoms of acute appendicitis in the setting of a DGH are often misattributed to strangulation symptoms with the correct diagnosis of acute appendicitis not usually obtained until surgical intervention. Bowel function has been reported as a potentially helpful clinical clue in differentiating an incarcerated femoral hernia from a de Garengeot hernia, as normal bowel function is retained in a DGH because only the appendix has herniated into the sac [11]. It has even been reported that, after the spontaneous reduction of a perforated appendix, the hernia neck seals off the infected collection, preventing peritoneal involvement [4]. Untreated symptomatic DGH may have severe complications including necrosis of hernia contents, perforation, sepsis, abscess formation, development of bowel obstruction, and necrotizing fascitis [10, 14]. Accurate diagnosis remains crucial with a reported case of appendicocutaneous fistula formation following misdiagnosis of DGHs as an abscess and subsequent surgical drainage [10].

The diagnosis of a DGH is difficult to make preoperatively, and only 4 reports of a preoperative CT diagnosis having been reported in the literature to date; herein, we present the fifth case [1, 4–6, 15]. In a review of DGHs by Kalles and colleagues, preoperative CT scanning was obtained in 9 patients; however, in only 4 cases was the CT diagnostic for a DGH [9, 11]. CT findings of a DGH can show the appendix within the hernia sac; and in the setting of acute appendicitis, inflammatory findings such as appendix dilatation, wall thickening, periappendiceal fat stranding, and a periappendiceal collection are shown. Additional CT findings in surgically proven cases of an incarcerated DGH include free fluid within the hernia sac, an engorged appendix with associated fat stranding, and extraluminal or intramural gas [3, 15]. The presence of intramural air in the absence of signs of bowel obstruction within an incarcerated hernia sac has been reported as a fairly specific sign for DGHs [2, 15]. Our case highlights the value in obtaining preoperative CT imaging, particularly with the ability to identify the appendix within the hernia sac and associated fluid collections as well. Although findings presented here are consistent with chronic appendicitis with superimposed acute inflammatory changes of the hernia sac, it can be inferred at some point that the appendix was in fact acutely inflamed.

It should be noted that the de Garengeot hernia should not be confused with the Amyand hernia which is an appendix containing inguinal hernia [3]. CT may also be used to differentiate a DGH from an Amyand hernia with Wechsler and colleagues suggesting that differentiation may be performed on the basis of the relationship between the hernia sac and pubic tubercle on CT images [16, 17]. The hernia sac extends medial to the pubic tubercles in all the incarcerated inguinal hernias, whereas the hernia sac is localized lateral to the pubic tubercles in all incarcerated femoral hernias [16]. Due to the close proximity of these structures, this may be difficult to ascertain on routine imaging, particularly in nonincarcerated cases [16].

Ultrasound findings of DGH can show the appendix as a blind-ending tubular structure surrounded by fluid and echogenic material within the hernia in the inguinal region [11]. As described by Filatov and colleagues, the relationship between the hernia and the femoral vasculature is important to establish for preoperative planning and diagnosis [11, 18, 19]. Magnetic resonance imaging (MRI) has been reported as an alternative imaging tool with the appendix identified as a blind-ending tubular structure arising from the right iliac fossa [9]. In the setting of acute appendicitis, the high intraluminal signal on T2-weighted sequences indicating intraluminal fluid and the presence of a susceptibility artifact on gradient echo sequences, indicating the presence of intramural air can be helpful [18]. MRI can provide several advantages over CT in diagnosing acute appendicitis, including high sensitivity for detecting inflammatory fluid surrounding the appendix (manifested as areas of high signal on T2-weighted sequences), absence of ionizing radiation, and lack of contrast administration [18].

Given the rarity of DGH, no standard approach to treatment has been described in the literature. There are several methods of surgical repair described in the literature including a Lockwood's infrainguinal, Lotheissen's transinguinal, and McEvedy's high incisions and laparoscopic repair [10]. In a review by Mizumoto et al. in 2016, they also describe the first ever use of the King's College approach, to successfully repair an incarcerated femoral hernia containing an appendix [10]. This single-incision technique allows for both femoral and inguinal hernia repair and permits access into the abdominal cavity, which is significant in cases of strangulated bowel or incarceration of the appendix [10]. Surgical approaches range from initial open drainage and interval appendectomy and hernia repair, to initial appendectomy followed by interval hernia repair [20]. It has been reported that if the groin was explored first, it was often not possible to reach the base of the appendix, and a subsequent laparotomy was necessary [20]. Several authors have reported that a normal appendix in the setting of a DGH does not need to be surgically excised and there have been several successful cases involving a simple reduction of the normal appendix followed by laparoscopic hernioplasty [3]. However, in cases with difficult reduction, or with clinical and imaging features suggestive of appendicitis or perforation, the risk of sepsis and abscess formation necessitate open appendectomy with herniorrhaphy or sutured repair [3].

The most common complication reported following DGH repair is wound infection, occurring in up to 29% of patients [8, 14]. Controversy exists regarding the use of foreign material in a contaminated field due to the risk of infection without a clear consensus regarding its use [8]. If there is no evidence of infection, some sources suggest that mesh repair may be performed [8]. Although there is a theoretical risk for infection with mesh repair, a few reports have mentioned successful mesh repair even in the presence of an inflamed appendix without evidence of postoperative infection [8]. In a comprehensive review by Mizumoto et al. in 2016, they suggested that the surgical approach should therefore be based on clinical judgment as well as the condition of the patient [10].

DGHs, although rare, should remain a consideration in elderly female patients presenting with inguinal pain. This case demonstrates the importance and value in obtaining preoperative imaging not only to aid in preoperative planning but to ensure the correct diagnosis and limit unexpected complications both in the operating room and postoperative setting.

## Figures and Tables

**Figure 1:** Axial contrast-enhanced CT images (a–d) demonstrate the appendix (solid arrows) entering into the right femoral hernia sac in keeping with a de Grangeot hernia. Within the hernia sac there is a fluid collection (dashed arrows) concerning for abscess or mucocele. Findings are confirmed on the sagittal reformatted image (e).

**Figure 2:** Coronal contrast-enhanced CT images demonstrate the appendix (solid arrows) entering into the right femoral hernia sac with surrounding periappendiceal fat stranding (dashed arrow) in keeping with chronic appendicitis.

**Figure 3:** (a) Hemotoxylin and eosinophilin staining at 4x magnification of the resected appendix demonstrating serosal congestion, edema, and fibrosis. (b) Hemotoxylin and eosinophilin staining at 4x magnification of the resected hernia sac adipose tissue demonstrating septal fibrosis and inflammation

**Table 1:** Retrospective review of the clinical features and outcomes in perforated appendix within a femoral hernia.

Report	Year	Patient age (years)	Gender	Duration of symptoms	Outcome
Waring [21]	1891	46	F	1 day (acute)	Uncomplicated
				2 years (chronic)	
Hodgson [22]	1925	70	F	8 months	Uncomplicated
Holiday and White [23]	1953	57	F	2 weeks	Uncomplicated
Carey [24]	1967	48	M	5 days (acute)	Wound infection
				5 months (chronic)	
Gerami et al. [25]	1970	71	M	5 months	Uncomplicated
Voitk et al. [26]	1974	59	F	15 years	Uncomplicated
		76	F	6 months	Death
Cuotolo et al. [27]	1978	73	F	14 days	Wound infection
Watkins [28]	1981	72	F	6 weeks	Uncomplicated
Rose and Cosgrove [29]	1988	72	F	1 week	Uncomplicated
		68	F	2 days	Uncomplicated
Guirguis et al. [30]	1989	80	F	5 days	Necrotizing fasciitis
Nguyen and Komenaka [31]	2004	88	M	2 days	Uncomplicated
D'Ambrosio et al. [4]	2006	71	F	2 weeks	Unknown
Piperos et al. [32]	2012	83	F	1 day	Uncomplicated
Hussain et al. [13]	2014	86	F	3 days	Uncomplicated
Ahmed et al. [9]	2014	71	M	3 days	Wound infection
Pritchard et al. [7]	2017	92	F	1 month	Wound infection
